# Optimal Diagnosis of COVID-19 Based on Convolutional Neural Network and Red Fox Optimization Algorithm

**DOI:** 10.1155/2021/4454507

**Published:** 2021-08-19

**Authors:** Ehsan Khorami, Fatemeh Mahdi Babaei, Aidin Azadeh

**Affiliations:** ^1^Department of Computer Engineering, Ravansar (Kermanshah) Branch, Islamic Azad University, Ravansar (Kermanshah), Iran; ^2^Department of Electrical and Computer Engineering, Mahallat Branch, Islamic Azad University, Mahallat, Iran; ^3^Shafaghkar Dena Technical Engineering Company, Ahvaz, Iran

## Abstract

SARS-CoV-2 is a specific type of Coronavirus that was firstly reported in China in December 2019 and is the causative agent of coronavirus disease 2019 (COVID-19). In March 2020, this disease spread to different parts of the world causing a global pandemic. Although this disease is still increasing exponentially day by day, early diagnosis of this disease is very important to reduce the death rate and to reduce the prevalence of this pandemic. Since there are sometimes human errors by physicians in the diagnosis of this disease, using computer-aided diagnostic systems can be helpful to get more accurate results. In this paper, chest X-ray images have been examined using a new pipeline machine vision-based system to provide more accurate results. In the proposed method, after preprocessing the input X-ray images, the region of interest has been segmented. Then, a combined gray-level cooccurrence matrix (GLCM) and Discrete Wavelet Transform (DWT) features have been extracted from the processed images. Finally, an improved version of Convolutional Neural Network (CNN) based on the Red Fox Optimization algorithm is employed for the classification of the images based on the features. The proposed method is validated by performing to three datasets and its results are compared with some state-of-the-art methods. The final results show that the suggested method has proper efficiency toward the others for the diagnosis of COVID-19.

## 1. Introduction

Coronaviruses are a large family of viruses that can cause disease in animals or humans. In humans, several types of viruses cause respiratory infections, from the common cold to more serious illnesses such as Middle East Respiratory Syndrome (MERS) and Severe Acute Respiratory Syndrome (SARS). A recently discovered virus from this family is SARS-CoV-2. It causes an infectious disease that has recently been discovered. The virus and its new disease were unknown before the outbreak in Wuhan, China, in December 2019.

People can get COVID-19 from other infected people with the virus. The disease can be spread from person to person with small drops in the nose or mouth when coughing or exhaling. These droplets land on objects and surfaces around a person. Other people then catch COVID-19 by touching these objects or surfaces and then touch their eyes, nose, or mouth. People can also get COVID-19 if they breathe in drops from a person with COVID-19 who coughs. This is why there has been emphasis on staying more than 1 meter (3 feet) away from someone who is sick. Medical imaging is a definitive way to diagnose coronaviruses, for example, CT scan of the lungs and chest X-ray images. Chest X-ray imaging exams are better types due to their valuable medical tool for a wide range of investigations. Chest X-ray imaging exams are a noninvasive and painless test that supports surgical and medical treatment planning to help experts in the diagnosis of the disease. The number of COVID-19 patients in the world is growing day by day. Based on the World Health Organization (WHO), infected patients of COVID-19 for April 17, 2021, are 140,888,075, and total death numbers until this date is 3,016,755 [1, 2].

One way of reducing the COVID-19 death rate and for avoiding the spread of this disease is to diagnose it in the initial stages. To provide a correct diagnosis system with high precision, chest X-ray imaging is an interesting method. The chest X-ray imaging as an early detection system can also increase the patients' survival chances.

Although X-ray imaging is typically one of the best imaging and nondestructive testing systems, some classes of the disease are not diagnosed by this method [3]. Therefore, offering a CAD-based computer-aided system can be used for efficient disease diagnosis [1]. Based on the literature, using computer-aided methods for the diagnosis of the disease is more efficient than that of physicians. Therefore, using these systems for helping physicians is a good technique to improve their accuracy.

Shorfuzzaman and Hossain [4] proposed a method based on artificial intelligence to better diagnose COVID-19 cases from chest X-ray (CXR) images. They utilized a synergistic methodology to participate in contrastive learning by a fine-adjusted ConvNet encoder for the detention of the unbiased feature representations to better diagnose COVID-19 cases. The performance of the suggested method was then validated based on two widely used datasets including normal, COVID-19, and pneumonia infected categories. The final results showed that the proposed model provides the highest accuracy against others in diagnosing COVID-19 from chest X-ray images.

Wu et al. [5] proposed a method based on Joint Classification and Segmentation (JCS) system to provide a real-time COVID-19 diagnosis system in chest CT scan images. The JCS system was trained by constructing a large-scale COVID-19 dataset. They also used lesion counts, opacification areas, and locations and thus benefit different aspects of diagnosis. Simulation results indicated that the suggested JCS diagnosis system has very well-organized results for COVID-19 detection.

Chen et al. [6] proposed a deep learning-based method for the automatic diagnosis of COVID-19. Contrastive learning of the study was utilized for encoder training to capture expressive feature representations on widely used lung datasets and the data is classified by the prototypical network. They authenticated the performance of the presented model compared with some other state-of-the-art methods. The results demonstrated the superiority of the proposed model toward the other comparative methods.

Zhang et al. [7] suggested a method based on deep learning for designing a detection system to determine COVID-19 from the chest X-ray concerning a consistent and fast diagnosis system. To provide the effectiveness of the model, ChestX-ray14 and GitHub repository 1 datasets were utilized. The final results indicated that the suggested technique gives better accurateness toward some state-of-the-art methods to show its superiority.

From the literature, it can be observed that several works were accomplished for the automatic diagnosis of COVID-19. However, literature shows that different kinds of methods have been proposed to develop a diagnosis system with higher efficiency. Also, using metaheuristic algorithms along with deep learning methods is scarce. This motivates us to work on this subject to assess how much this combination can be useful for the diagnosis of COVID-19. In this study, a new CAD-based system is utilized for the diagnosis of COVID-19 in chest X-ray images. Here, an optimized deep network based on a newly introduced metaheuristic, called Red Fox Optimization (RFO) algorithm, is employed for this purpose.

## 2. Image Preprocessing

Preprocessing is the process of improving the quality of an input image. The image preprocessing of medical images is vital to remove cases like noise or light. In medical images, some disturbances have been made due to their high-frequency reception, different brightness in the field, and problems with distant orientation. This can be corrected by artificial intelligent [8]. So, after medical image acquisition, the preprocessing operations should be accomplished to remove noise and develop the areas differentiation.

### 2.1. Contrast Enhancement

Contrast enhancement of an image is a process to facilitate the interpretation and understanding of images. During the image processing, it may not have enough resolution or the desired quality to display the information in the images. For this reason, each image may require special adjustments in terms of brightness and scatter [9]. Image processing and artificial intelligence are also used for medical imaging purposes [10]. This study uses contrast enhancement to highlight the lung areas on the images with no changes on the other areas. Here, 16-bit Lookup Table is used to develop the contrast of the image. This technique is accomplished by Lookup Table based on the following equation [11]:

(1) $$\begin{array}{c} y_{hist}=\frac{x_{\text{hist}}-{\text{Min}}_{\text{hist}}}{{\text{Max}}_{\text{hist}}-{\text{Min}}_{\text{hist}}}, \end{array}$$

where Min_hist_ and Max_hist_ stand for the lowest and the highest levels of the gray magnitudes for the main image histogram, respectively, and *x*_hist_ and *y*_hist_ describe the input image before and after contrast enhancement, respectively.

### 2.2. Data Normalization

Data normalization is used to change the scale in most multivariate methods and techniques. Thus, in addition to the impact of the size of the variable criterion, all variables are important in terms of weights or coefficients created by the model. One method of resizing data is to use the min-max normalization method. In this way, in addition to unifying the data scale, the edges of their change will also be in the range [0, 1]. This calculation method is often used when we want to determine the degree of similarity between points. Suppose *A* as data that should be mapped from the dataset between *A*_min_ to *A*_max_. For this purpose, we have the following equation [12]:

(2) $$\begin{array}{c} A_{\text{normalized}}=\frac{A-A_{\min}}{A_{\max}-A_{\min}}. \end{array}$$

The reason for using min-max normalization here is that it guarantees all features to be exacted in the same scale.  Figure 1 shows some examples of image processing on the input images.

## 3. Image Segmentation

The Otsu thresholding method along with mathematical morphology is used here to determine the region of interest (ROI). The Otsu method offers a low-cost segmentation to provide a method with less complexity.

The Otsu method works based on intergroup variance optimization and decreasing pixels' intragroup variance to automatic segmentation of the input images. Global thresholding has some problems during the times when the image background resolution is not enough (heterogeneity effect). For refining this effect, the local thresholding method is used [13]. Based on the Otsu thresholding method, the threshold value is examined that minimizes the class-in-between variance. This is done based on the following equation [14]:

(3) $$\begin{array}{c} \sigma_{\omega }^{2}\left(t\right)=\omega_{1}\left(t\right)\sigma_{1}^{2}\left(t\right)+\omega_{2}\left(t\right)\sigma_{2}^{2}\left(t\right), \end{array}$$

where *ω*_*i*_ represents the probability in two separated groups with a magnitude equal to *t* and *σ*_*i*_^2^ describes the value of the variance within the groups.

In other words, the Otsu method specifies that the class variance minimization is equal to variance maximization in class-within; in other words,

(4) $$\begin{array}{c} \sigma_{b}^{2}\left(t\right)=\sigma^{2}-\sigma_{\omega }^{2}\left(t\right)=\omega_{1}\left(t\right)\omega_{2}\left(t\right){\left[\mu_{1}\left(t\right)-\mu_{2}\left(t\right)\right]}^{2}, \end{array}$$

where *μ*_*i*_ represents the mean value. The pseudocode of the Otsu algorithm is given in Algorithm 1.

Afterward, three postprocessing techniques based on mathematical morphology are used to improve the segmentation accuracy. The three steps are using mathematical filling, closing, and opening [15]. To do so, extra holes in the images have been first filled using a mathematical filling. The mathematical model of this operator is as follows:

(5) $$\begin{array}{c} X_{k}=\left(X_{k-1}⊕B\right)\cap A^{c},\;k=1,2,3\ldots , \end{array}$$

where *A* and *B* represent the processed area and the constructing element, respectively.

The next process is to use the mathematical opening to remove the useless low-cost information with no changes on the other parts of the image. The mathematical opening is modeled as follows:

(6) $$\begin{array}{c} A\circ B=\left(A⊖B\right)⊕B. \end{array}$$

Finally, mathematical closing is utilized to connect the narrow parts by the following equation:

(7) $$\begin{array}{c} A\cdot B=\left(A⊕B\right)⊖B. \end{array}$$

This study uses 3 × 3 identity matrix as a structuring element.  Figure 2 shows some examples of total image segmentation to determine the ROI in chest X-ray images.

## 4. Feature Extraction

Although machine vision techniques are widely used to extract features, these techniques cannot be used in some images, such as medical images. In recent years, much attention has been paid to various areas of image processing and computer vision. To extract the properties of images, especially medical images, it is necessary to extract the features of color, extract the texture, determine the homogeneity of the image, and filter to improve the output. Before performing the recovery operation, all the required features for the image database must be extracted. For reducing the complexity of the processing, the image features are extracted instead of using pixel values. In this study, Discrete Wavelet Transform (DWT) and the gray-level cooccurrence matrix (GLCM) have been used for this purpose.

### 4.1. Discrete Wavelet Transform (DWT)

Wavelet Transform is one of the most important mathematical transformations used in various fields of science. The main idea of wavelet transform is to overcome the weaknesses and limitations of the Fourier transform. Unlike Fourier transform, this conversion can also be used for nonstatic signals and dynamic systems.

Several kinds of DWT models have been proposed for different applications. One of the widely used methods for medical image feature extraction is to use multiresolution analysis (MRA). In MRA, the DWT implementation is accomplished using a series of uninterrupted operations where each part contains signal filtering and downsampling. On each step, the signal content has been decomposed into two orthogonal subspaces containing a low-pass filter (LL) and a high-pass (HH) filter [16], which is then divided into four segments: LH, LL, HH, and HL. To provide a high-resolution frequency, this decomposition has rendered successively, so that the approximation signal has been passed over a pair of high- and low-pass filters and decomposed into two new approximate and information signals. Then, the read speed was reduced to 50%. To offer more information, the HL subbands with more efficiency have been performed. This is mathematically expressed as follows [17]:

(8) $$\begin{array}{c} P_{\text{dwt}}\left(s\right)=\left\{\begin{array}{c} d_{i,j}=\sum f\left(s\right)\times H*i\left(s-2\times i\times j\right),\\ d_{i,j}=\sum f\left(s\right)\times L*i\left(s-2\times i\times j\right), \end{array}\right) \end{array}$$

where *d*_*i*,*j*_ describes the feature of the component in signal *f*(*s*), *L* and *H* represent the low-pass filter coefficient and the high-pass filter coefficient, respectively, and *i* and *j* provide the translation and the wavelet factors scales, respectively.

### 4.2. Gray-Level Cooccurrence Matrix

Gray-level cooccurrence matrix (GLCM) is one of the statistical methods of tissue extraction proposed by Haralick in 1973. This method is based on the distance and angle between two pairs of pixels located in a window with specific dimensions to calculate vectors features. This matrix consists of *G* × *G* arrays, each of which is equal to *Pd*, where *d*=(d*x*, d*y*) describes the displacement vector, i.e., [18]

(9) $$\begin{array}{c} P_{d}\left(i,j\right)=\left|\left[\left(\left(r,s\right),\left(t,v\right)\right):I\left(r,s\right)=i,I\left(t,v\right)=j\right]\right|, \end{array}$$

where

(10) $$\begin{array}{c} \left(r,s\right),\left(t,v\right)\in N\times N,\;\;\left(t,v\right)=\left(r+\text{d}x,s+\text{d}y\right), \end{array}$$

and |.| describes the dimension of the set.

This matrix can be applied to the whole image or any area of it. To extract texture features, we must assign a number to each pixel of the image. So, we first put individual windows on each pixel, and in this window, we calculate the GLCM. Then, using this matrix, a large number of texture features can be extracted using statistical relationships, with each property assigning a number to each pixel. Among the most important properties from the GLCM, second angular momentum, contrast, inverse differential torque, irregularity, correlation, and autocorrelation have been considered.

This study uses a radial distance of 1 with four zero angles and several 256 gray surfaces. Among these features, homogeneity provides a local uniformity feature to generate multiple/single intervals for accusing the nontextured/textured characteristics; entropy determines the image selected interference; contrast determines the pixels intensity magnitude and their neighborhood; correlation states the spatial features dependence among the pixels; and energy defines the repetitive pixel pairs quantity. The miasmatical formulation of these methods is given below:

(11) $$\begin{array}{c} \text{Homogeneity}=\overset{m-1}{\underset{i=0}{\sum }}\overset{n-1}{\underset{j=0}{\sum }}\frac{1}{1+{\left(i-j\right)}^{2}}f\left(i,j\right),\\ \text{Entropy}=-\overset{m-1}{\underset{i=0}{\sum }}\overset{n-1}{\underset{j=0}{\sum }}\log_{2}\;f\left(i,j\right),\\ \text{Contrast}=\overset{m-1}{\underset{i=0}{\sum }}\overset{n-1}{\underset{j=0}{\sum }}{\left(i-j\right)}^{2}f\left(i,j\right),\\ \text{Correlation}=\frac{\sum_{i=0}^{m-1}\sum_{j=0}^{n-1}\left(i,j\right)f\left(i,j\right)-\mu_{i}\mu_{j}}{\sigma_{i}\sigma_{j}},\\ \text{Energy}=\sqrt{\overset{m-1}{\underset{i=0}{\sum }}\overset{n-1}{\underset{j=0}{\sum }}f^{2}\left(i,j\right)}. \end{array}$$

After extracting the features based on the GLCM and DWT, they have been injected into a classifier for the final diagnosis. The present study uses Convolutional Neural Network (CNN) as a second-order statistic to reflect the overall average for the degree of correlation between pairs of pixels in different aspects (in terms of homogeneity, uniformity, etc.).

## 5. Classification

### 5.1. Convolutional Neural Networks

Convolutional Neural Networks (CNNs) are deep types of neural networks that extended into three dimensions for increasing system efficiency. These types of neural networks are specially introduced for image processing applications.

Convolutional Neural Networks contain three main layers including the convolutional layer, pooling layer, and the fully connected layer. Each layer has a special duty. This is accomplished during two steps: feedforward and backward for preparation. At first, the features are injected into the network which is done by point multiplication between the input features and the variables of the neurons and the application of convolution operations in the layers.

Afterward, the network output has been evaluated. To accomplish the variables related to network training, network output results have been performed to evaluate the network error rate. To do this end, a comparison between the output of the network and the optimal solution has been performed. Then, by using the achieved error ratio, the postrelease phase has been started. The chain rule is used to achieve the gradient value of the variables and update them. The next step is feedforward. This phase continues until the network is prepared for application. The purpose of CNN in this research is to use it as a classifier of the features entered from the previous section in chest X-ray images for COVID-19 diagnosis. To give optimum weighting among network connections, the backpropagation technique is utilized and the activation mechanism is chosen rectified linear unit (ReLU). Size reduction of the output is based on max pooling and the cross-entropy loss reduction is based on the gradient descent method. The backpropagation process is modeled below:

(12) $$\begin{array}{c} L=\overset{N}{\underset{j=1}{\sum }}\overset{M}{\underset{i=1}{\sum }}-d_{j}^{\left(i\right)}\log\;z_{j}^{\left(i\right)},\;d_{j}=\left(0,\ldots ,0,\underset{k}{\underset{︸}{1,\ldots ,1}},0,\ldots ,0\right), \end{array}$$

where *d*_*j*_ defines the desired output vector and *z*_*j*_ describes the obtained output vector for the *m*^th^ class. The Softmax function is mathematically modeled as follows:

(13) $$\begin{array}{c} z_{j}^{\left(i\right)}=\frac{e^{f_{j}}}{\sum_{i=1}^{M}e^{f_{i}}}, \end{array}$$

where *M* represents the number of samples.

To provide a function with higher values, a weighting penalty (*ρ*) has been used as follows:

(14) $$\begin{array}{c} L=\overset{N}{\underset{j=1}{\sum }}\overset{M}{\underset{i=1}{\sum }}-d_{j}^{\left(i\right)}\log\;z_{j}^{\left(i\right)}+\frac{1}{2}\rho \underset{K}{\sum }\underset{L}{\sum }W_{k,l}^{2}, \end{array}$$

where *W*_*k*_ describes the connections weight and *L* and *K* represent the total numbers of layers and the layer *l* connections, respectively.

The layouts of CNN are usually defined by trials and errors that present imprecise results. Several automated and optimized works are accomplished to address this issue [19]. Among different types of methods for solving this issue, metaheuristic algorithms are so popular. This study uses one of the newest metaheuristic techniques, called Red Fox Optimizer, to provide an effective CNN based on the previously described cases. The main advantage of CNN compared to its predecessors is that it automatically detects the important features without any human supervision.

### 5.2. Red Fox Optimizer (RFO)

As mentioned before, for optimal diagnosis of COVID-19 based on CNN, an optimization tool is required. To obtain the optimum solution of a problem, it should be minimized or maximized (in this study, a minimization process is required) [20]. Different methods are introduced to achieve the optimal solutions [21]. The Karush–Kuhn–Tucker technique (KKT), Hamiltonian technique, and other classic techniques have an important benefit [22]. Also, these methods can achieve the exact solution for the problem, but there is a major deficiency: these methods often cannot find a solution for complex nonlinear problems. Metaheuristics are presented as new optimization techniques to solve these problems [23, 24]. These approaches can find a solution for all types of problems by obtaining a pseudooptimum solution. The metaheuristics are inspired by different phenomena such as behaviors of humans and animals contest to hunt [25]. Different kinds of these algorithms are introduced, for example, Grasshopper Optimizer (GO) [26], Cuckoo Optimizer (CO) [27], Harris Hawks Optimizer (HHO) [28], and Mayfly Optimizer [29].

Foxes are small to medium-sized, omnivorous mammals belonging to several genera of the family Canidae; due to their long, slender legs, pointed noses, thick tails, and slender limbs, foxes are distinguished from other family members or big dogs. The lifestyle of this animal is very social and thus it has flexible behavior. They can be seen all over the world with different diets. Their habitats are polar regions, deserts, and treeless plains. This animal is a type of populated fox species with great distribution. The foxes are small and fast animals that can hunt the prey while taking care about the other risks. Also, they are well-known because of their adaptability and higher intelligence. These types often chose one of two lifestyle types. In one lifestyle, they always live in a crew in a position with considering a territory [30–32]. In the second lifestyle, they live in a nomadic crew. The leader is an alpha couple in both ways of life. After enough growth of young individuals in each crew, they decide to leave or to stay with the crew.

The Red Fox Optimizer (RFO) is a new metaheuristic optimization algorithm that is inspired by the hunting lifestyle among the red foxes. When hunting, the red fox gets close to the prey gradually whereas it hides behind the bushes, and after, the prey is unexpectedly attacked. Similar to other metaheuristics, the RFO algorithm includes exploitation and exploration.

By the fox prey choice at faraway locations from the prey, the exploration term is defined, and the exploitation term is defined based on nearing the fox to the prey wherever possible to attack the prey. The RFO initialization is modeled by random individual generation as follows:

(15) $$\begin{array}{c} X=\left[x_{0},x_{1},\ldots ,\;x_{n-1}\right], \end{array}$$

where *i* denotes the number of population, (*X*_*j*_^*i*^)^*t*^ describes the *x*_*i*_ in iteration  *t*, and *j* is the problem dimension in the searching space.

With assuming *f* as condition function in *R*^*n*^ where *n* stands for the parameters in the range [*a*, *b*]^*n*^,

(16) $$\begin{array}{c} {\left(X\right)}^{i}=\left[{\left(x_{0}\right)}^{i},{\left(x_{1}\right)}^{i},\ldots ,\;{\left(x_{n-1}\right)}^{i}\right], \end{array}$$

where *a*, *b* ∈ *R*.

Thus, the optimum solution is achieved while *f* ((*X*)^*i*^) suggests the global optimal. Individuals are assumed as a certain assignment to help the crew for exploration.

If the area does not include adequate prey, the individuals move to another region to get a better chance for prey. The location is shared with the others if there is a more proper region obtained. Therefore, the individuals were adapted based on the cost value. Squared Euclidean distance is applied in this regard, i.e.,

(17) $$\begin{array}{c} D\left({\left({\left(X\right)}^{i}\right)}^{t},{\left(X_{\text{best}}\right)}^{t}\right)=\sqrt{{\left({\left(X\right)}^{i}\right)}^{t}-{\left(X_{\text{best}}\right)}^{t}}. \end{array}$$

Therefore, all candidates migrate by the optimum solution as follows:

(18) $$\begin{array}{c} {\left({\left(X\right)}^{i}\right)}^{t}={\left({\left(X\right)}^{i}\right)}^{t}+\alpha \times \mathrm{sgn}\left({\left(X_{\text{best}}\right)}^{t}-{\left({\left(X\right)}^{i}\right)}^{t}\right), \end{array}$$

where *α* is a random value.

Here, the new location of the candidates should suggest a proper solution. If not so, the previous location will have remained. When the red fox observes the prey, it gets close to the prey. It is defined as the exploitation of the Red Fox Optimization algorithm, which is modeled by assuming a random value *r* in the range [0, 1]:

(19) $$\begin{array}{c} \left\{\begin{array}{cc} \text{move closer} & \text{if }r>\frac{3}{4},\\ \text{stay and hide} & \text{if }r\leq \frac{3}{4}. \end{array}\right) \end{array}$$

Afterward, an enhanced cochleoid formula is used to figure out the member's motion.

The next term is conditioned by a variable, defined as radius, which is based on two variables: *a* which is a random value in the range [0, 0.2] and the variable *ϕ*_0_ which denotes a value in the range [0,2*π*] that defines the fox observation angle. Mathematically, this term can be modeled as follows:

(20) $$\begin{array}{c} r=\left\{\begin{array}{cc} a\times \frac{\sin\left(\phi_{0}\right)}{\phi_{0}}, & \text{if }\phi_{0}\neq 0,\\ \gamma , & \text{if }\phi_{0}=0, \end{array}\right) \end{array}$$

where *γ* represents a random value between 0 and 1. Mathematically, the fox population nearing the prey is modeled as follows:

(21) $$\begin{array}{c} \left\{\begin{array}{c} x_{0}^{\text{New}}=a\times r\times \;\cos\left(\phi_{1}\right)+x_{0}^{\text{actual}}\\ x_{1}^{\text{New}}=a\times r\times \;\sin\left(\phi_{1}\right)+a\times r\times \;\cos\left(\phi_{2}\right)+x_{1}^{\text{actual}}\\ x_{1}^{\text{New}}=a\times r\times \;\sin\left(\phi_{1}\right)+a\times r\times \;\sin\left(\phi_{2}\right)+a\times r\times \;\cos\left(\phi_{3}\right)+x_{2}^{\text{actual}}\\ \vdots \\ x_{n-1}^{\text{New}}=a\times r\times \overset{n-2}{\underset{k=1}{\sum }}\sin\left(\phi_{1}\right)+a\times r\times \;\cos\left(\phi_{n-1}\right)+x_{n-2}^{\text{actual}}\\ x_{n-1}^{\text{New}}=a\times r\times \;\sin\left(\phi_{1}\right)+a\times r\times \;\sin\left(\phi_{2}\right)+\cdots +a\times r\times \;\sin\left(\phi_{n-1}\right)+a\times r\times \;\sin\left(\phi_{n-1}\right)+x_{n-a}^{\text{actual}}. \end{array}\right) \end{array}$$

In the created population, 5% of the worst members are eliminated and several new members were included to the individuals to have fixed size of the population. Likewise, two optimum members were achieved as (*X*(1))^*t*^ and (*X*(2))^*t*^ as alpha couple in iteration *t*. Then, the territory center is obtained as given below:

(22) $$\begin{array}{c} H_{c}^{t}=\frac{1}{2}{\left(X\left(1\right)\right)}^{t}-\;{\left(\text{X}\left(2\right)\right)}^{t}, \end{array}$$

and the territory diameter by Euclidean distance is defined as follows:

(23) $$\begin{array}{c} H_{d}^{t}=\sqrt{{\left(X\left(1\right)\right)}^{t}-\;{\left(\text{X}\left(2\right)\right)}^{t}}. \end{array}$$

A random amount, *σ*, is chosen in this process that is between 0 and 1:

(24) $$\begin{array}{c} \left\{\begin{array}{cc} \text{New nomadic candidate,} & \text{if }\sigma >0.45,\\ \text{Reproduction of the alpha couple,} & \text{if }\sigma \leq 0.45. \end{array}\right) \end{array}$$

Random locations are obtained in the searching space. Then, the new members are set up by the alpha couple, i.e.,

(25) $$\begin{array}{c} {\left(X^{\text{rep}}\right)}^{t}=\frac{\sigma }{2}{\left(X\left(1\right)\right)}^{t}-\;{\left(X\left(2\right)\right)}^{t}. \end{array}$$

The utilized parameters for RFO in this study are as follows:  *a*=0.2 and *ϕ*_0_=1.

### 5.3. Hybrid RFO and CNN for Classification

The classification is one of the most important parts of each medical imaging. After features extraction, they should be injected into a classifier for diagnosing the disease. Based on the explanations above, CNN uses the backpropagation technique for learning. This study developed an RFO algorithm for the proper selection of network weights in CNN by minimizing the mean square error (MSE). The MSE can be mathematically defined as follows:

(26) $$\begin{array}{c} \text{MSE}=\frac{1}{T}\overset{L}{\underset{j=1}{\sum }}\overset{M}{\underset{i=1}{\sum }}{\left(y_{j}^{i}-d_{j}^{i}\right)}^{2}, \end{array}$$

where *M* and *L* describe the output value of the layers and the data, respectively, and *y*_*j*_^*i*^ and *d*_*j*_^*i*^ represent the achieved and the proper magnitudes for *j*^th^ unit in the output layer of the network in time *t*, respectively.

## 6. Results and Discussions

The proposed method proposes an effective automated method for automatic diagnosis of the COVID-19 based on hybridizing the convolutional neural network and Red Fox Optimization algorithm. The method is a pipeline technique including preprocessing, segmentation, features extraction, and finally classification.  Figure 3 shows the block diagram of the proposed system.

### 6.1. Dataset Description

To validate the effectiveness of the proposed method, it should be testified on a standard COVID-19 dataset. There are different types of datasets for COVID-19. In this study, consistent resources were collected by the Renmin Hospital of Wuhan University and two affiliated hospitals (the Third Affiliated Hospital and Sun Yat-Sen Memorial Hospital) of the Sun Yat-Sen University in Guangzhou with 76 and 12 patients employed [33].  Figure 4 shows some examples of the employed chest X-ray images for the analysis.

### 6.2. Simulations

After implementing the Discrete Wavelet Transform on the ROU in input chest X-ray images based on LL and HL decomposition characteristics, the GLCM features of these decompositions have been obtained. Afterward, the obtained features have been injected into the proposed CNN-AOA classifier for the final diagnosis. Here, five features including correlation (Cr), homogeneity (*H*), energy (E), entropy (ER), and contrast (CN) have been employed for applying into the LL and the HL subband levels on the image.  Table 1 reports the feature extraction of the training data.

The feature extraction of the testing data is also reported in Table 2.

To provide proper analysis on the suggested methodology, it has been verified using three measurement indicators including sensitivity, specificity, and precision. The mathematical formulation of these three indicators is given below:

(27) $$\begin{array}{c} \text{specificity}\left(\%\right)=\frac{\text{TN}}{\text{FP}+\text{TN}},\\ \text{sensitivity }\left(\%\right)=\frac{\text{TP}}{\text{TP}+\text{FN}},\\ \text{accuracy}\left(\%\right)=\frac{\text{TP}+\text{TN}}{\text{TP}+\text{FP}+\text{FN}+\text{TN}}, \end{array}$$

where TN and TP are true negative and true positive and FN and FP represent false negative and false positive, respectively. The suggested method has been compared with 3 state-of-the-art methods and the results are shown in Figure 5. The methods are as follows: the method of Aminu [34], Wu et al. method [5], and Singh et al. method [35].

According to Figure 5, the proposed RFO-CNN classifier with 95.60% accuracy provides the highest accuracy among the comparative methods, and Aminu's, Wu's, and Singh's methods with 84.56%, 84.29%, and 83.34%, respectively, are in the next ranks. In addition to accuracy, the specificity of the suggested method with 69.14% provides the best achievements compared to the other methods. Specificity shows how well it can separate the disease from the healthy cases. Here, Wu's method with 49.38% specificity is in the next rank and Aminu's and Singh's methods with 44.08% and 36.09% are in the next ranks. At last, sensitivity is a fundamental characteristic of diagnostic imaging tests which shows how well it can be positive among all those with the condition. Here, the proposed method with 97.47% sensitivity has the best results, and Singh's, Aminu's, and Wu's methods with 96.58%, 93.76%, and 88.59%, respectively, are in the next ranks. Finally, the results showed the higher efficiency of the system for usage as a proper system for COVID-19 diagnosis.

## 7. Conclusions

COVID-19 is a new member of coronaviruses named by the World Health Organization (WHO) on February 11, 2020, based on the year of its outbreak and its infectious agent. Recently, several types of research works were introduced on chest X-ray images to diagnose this disease with high accuracy based on image processing and computer vision. In the present research, a new pipeline methodology was proposed for the automatic diagnosis of COVID-19. At first, the input chest X-ray images were preprocessed based on contrast enhancement and data normalization to improve the input image quality and shift them into a standard interval. Then, simple image segmentation is followed by mathematical morphology. To provide the main features of the chest X-ray images, a combined gray-level cooccurrence matrix (GLCM) and Discrete Wavelet Transform (DWT) were established on the segmented images. Finally, the Red Fox Optimization algorithm was performed to a Convolutional Neural Network (CNN) for the final classification of the features. Experimental results were compared with three other state-of-the-art methods to indicate the method's efficacy. The results showed that although the proposed method is efficient for this purpose, it needs much time for the analysis (i.e., higher time complexity). Therefore, in future work, the main focus should be on determining a method for improving the system to decrease its time complexity.

## Figures and Tables

**Figure 1:** Some examples of image processing on the input images.

**Figure 2:** Some examples of image segmentation on the preprocessed images.

**Figure 3:** The block diagram of the proposed system.

**Figure 4:** Some examples of COVID-19 chest X-ray images.

**Figure 5:** The comparison analysis between the proposed method and the studied methods applied to the chest X-ray images dataset.

**Algorithm 1:** The pseudocode of the Otsu algorithm.

**Table 1:** The feature extraction of the training data.

#	*H*	CR	*E*	CN	ER
1	0.720	0.056	0.788	0.311	0.311
2	0.840	0.174	0.973	0.052	0.275
3	0.832	0.039	0.889	0.029	0.295
4	0.807	0.038	0.905	0.027	0.407
5	0.764	0.035	0.974	0.116	0.413
6	0.836	0.064	0.897	0.010	0.228
7	0.613	0.068	0.984	0.043	0.306
8	0.788	0.006	0.941	0.028	0.386
9	0.612	0.073	0.986	0.030	0.319
10	0.715	0.037	0.974	0.053	0.427

**Table 2:** The feature extraction of the testing data.

#	*H*	CR	*E*	CN	ER
1	0.812	0.066	0.802	0.051	0.286
2	0.761	0.057	0.873	0.015	0.329
3	0.804	0.040	0.847	0.053	0.353
4	0.842	0.032	0.806	0.022	0.211
5	0.767	0.030	0.672	0.017	0.412
6	0.659	0.034	0.789	0.033	0.400
7	0.783	0.019	0.906	0.064	0.336
8	0.702	0.026	0.843	0.040	0.438
9	0.635	0.037	0.822	0.052	0.452
10	0.736	0.072	0.946	0.082	0.369

## Data Availability

In this study, consistent resources were collected by the Renmin Hospital of Wuhan University and two affiliated hospitals (the Third Affiliated Hospital and Sun Yat-Sen Memorial Hospital) of the Sun Yat-Sen University in Guangzhou with 76 and 12 patients employed that can be achieved by emailing to these places.
